RETRACTED

# Oxytocin versus a combination of tranexamic acid and ethamsylate in reducing intraoperative bleeding during abdominal myomectomy: a randomized clinical trial

**DOI:** 10.1186/s12905-023-02549-z

**Published:** 2023-07-29

**Authors:** Ahmed Mahmoud Abdou, Elsayed Eldesouky, Elsayed Farag, Attia Mohammed, Doaa Fathy Mohamed Abdelaziz, A. Shaaban, Mostafa Ellaban, Abd Elhalim Mohamed Abd Elhalim, Ahmed Gamal Abo Elsror, Alrefaai Abd Elfattah Marai, Faiza Abdel-Hakam, Mohamed Abd-ElGawad, Asmaa Ahmed Elrashedy, Hanaa Abdelmonem, Mohamed Abdelmonem Kamel, Ibtesam K. Afiffi, Hazem Galal Abdelhameed Elsayed, Sameh Abdelmoneim Abdelhamed, Almandouh H. Bosilah, Heba Marie

**Affiliations:** 1 Obstetrics and Gynecology, Faculty of Medicine, Zagazig University, Zagazig, Egypt; 2 Department of Obstetrics and Gynecology, Faculty of Medicine, Alazhar University in Cairo, Cairo, Egypt; 3 Department of Obstetrics and Gynecology, Alazhar University for Girls in Cairo, Cairo, Egypt; 4 Department of Obstetrics and Gynecology, Faculty of Medicine, Alazhar University in Assuit, Assuit, Egypt; 5 International Islamic Institute for Studies and Population Research Alazhar University in Cairo, Cairo, Egypt; 6 MBBCh, Faculty of Medicine Fayoum University, Fayoum, Egypt; 7 Faculty of Medicine, Kafr El-Shaikh University, Kafr El-Shaikh, Egypt; 8 Department of Medical Microbiology and Immunology, Faculty of Medicine, Tanta University, Tanta, Egypt; 9 Department of Basic &Clinical Oral Sciences &, Faculty of Dental Medicine, Umm Al-Qura University, Makkah, Saudi Arabia; 10 Department of Obstetrics and Gynecology, Faculty of Medicine, Fayoum University, Fayoum, Egypt; 11 Department of Obstetrics and Gynecology, Faculty of Medicine, Damiata University, Damiata, Egypt; 12 Department of Obstetrics and Gynecology, Faculty of Medicine, Cairo University, Cairo, Egypt

**Keywords:** Abdominal myomectomy, Blood loss, Oxytocin, Ethamsylate, Tranexamic acid

## Abstract

**Objective:**

Myomectomy is the preferred surgical approach to manage uterine fibroids. However, uterine fibroids are highly vascular tumors and, consequently, extremely susceptible to problems from myomectomy-related hemorrhage. Hence, we aim to compare oxytocin efficacy and safety profile versus tranexamic acid (TA) with ethamsylate for reducing bleeding during myomectomy.

**Methods:**

This randomized, double-blinded multicenter study was performed between 20^th^ August 2020 and 20^th^ October 2020 at El-Galaa Teaching Hospital, El Hussein University Hospital, Al-Azhar University Hospitals of Assiut, and Al-Azhar University Hospitals of Damietta. One hundred and eighty patients were enrolled and divided into three groups: group (1) received an injection of 30 IU of oxytocin in 500 ml of normal saline; group (2) received injections of 1 g of TA, 250 mg of Ethamsylate, and 110 ml of normal saline IV; and group (3) received an injection of 110 ml of normal saline IV just before surgical incision.

RETRACTED

**Results:**

In 180 premenopausal women, oxytocin and TA with ethamsylate had no significant value in lowering intraoperative blood loss compared with the placebo for abdominal myomectomy (666.25 ± 183.03, 630.72 ± 145.83, and 646.67 ± 168.92, respectively (*P* = 0.506)). Non-significant trends were observed for a reduction in operation time (*P* = 0.760), intra/postoperative blood transfusion (*P* = 0.624), hospital stay (*P* = 0.986), postoperative fever (*P* = 0.659), and wound infection (*P* = 1).

**Conclusion:**

Oxytocin and TA with ethamsylate had no significant value in lowering intraoperative blood loss compared with the placebo for abdominal myomectomy which opens a new question about the role of the use of the hemostatic drug during myomectomy especially in centers with limited resources and had higher rates.

**Trial registration:**

The study was registered on Pan African Clinical Trials Registry with the following number: PACTR202008739887429 and was approved on 24/08/2020.

## Background

With about 235 million women affected globally [1], uterine fibroids, also termed leiomyomas, are the most common benign tumors of the female genitalia [2]. Recent population-based statistics show that the prevalence of fibroids gradually rises throughout the childbearing age (maximum incidence at the age of 50) and is more prominent in low-parity women of the black race [3].

Clinically, uterine fibroids are frequently asymptomatic, but in 30% of cases, fibroids can be symptomatic and cause various critical complications. These complications include pelvic pain, heavy menstruation, anemia, frequent urination, bowel problems, and infertility [2].

The current management options for fibroids include surgical, radiological, and pharmaceutical management [2]. The surgical option is the most frequently chosen when pharmacological treatments fail to manage the condition. Myomectomy is the preferred surgical approach of choice, particularly for people who want to keep their uterus for fertility problems [4].

Regardless of the myomectomy approach, uterine leiomyomas are highly vascular tumors [5] and, consequently, extremely susceptible to problems from myomectomy-related hemorrhage [6]. Additionally, myomectomy is not a risk-free treatment, and the most often reported consequence is intraoperative blood loss, which can go excessive enough to necessitate an immediate blood transfusion [7]. Furthermore, life-threatening hemodynamic instability, shock, coagulopathy, and mortality are potential consequences if the bleeding is not effectively controlled following myomectomy. Thus, measures to minimize bleeding and associated morbidities are essential to lower morbidity and mortality during myomectomy [8].

RETRACTED

Few trials have looked at the effectiveness of various perioperative pharmacologic treatments, such as oxytocin, tranexamic acid (TA), and ethamsylate, to reduce blood loss and associated morbidities during myomectomy [8].

Oxytocin is one of the hormones that the pituitary gland is their primary source of secretion, as its primary role is to cause uterine contractions during childbirth. For preventing postpartum hemorrhage, oxytocin is the drug of preference [9]. Thus, its intraoperative administration can efficiently reduce blood loss during abdominal myomectomy [10].

TA is a manufactured version of the human amino acid lysine. Its mechanism of action is reducing through its antifibrinolytic action as it inhibits plasminogen from being transformed into plasmin [11]. On the other hand, ethamsylate prevents capillary bleeding. It affects the first stage of hemostasis by enhancing platelet adhesiveness and regaining capillary resistance which has a hemostatic impact. It accelerates platelet aggregation and cuts down on bleeding time. Whenever there are enough platelets, it lessens capillary bleeding. The medication increases capillary wall stability and inhibits hyaluronidase [12]. Hence, based on their mechanism of action, the combination of TA and ethamsylate seems promising to reduce the bleeding tendency during abdominal myomectomy. Thus, we conducted this randomized controlled trial (RCT) to compare oxytocin efficacy and safety profile versus TA with ethamsylate for reducing blood loss during myomectomy.

## Methods

### Study design and study population

We followed the CONSORT reporting guidelines in reporting our randomized, double-blinded multi-center study which was performed between 20^th^ August 2020 and 20^th^ October 2020 at El-Galaa Teaching Hospital, El Hussein University Hospital, Al-Azhar University Hospitals of Assiut, and Al-Azhar University Hospitals of Damietta. All participants provided informed consent before enrollment and the study was approved by the Ethical Committee of Quality Education Assurance Unit of the Al Azhar Faculty of Medicine. On 28/8/2020, the study's protocol was accepted by the Pan African Clinical Trials Registry under the number PACTR202008739887429. The study was performed according to the Declaration of Helsinki.

We included premenopausal women between the ages of 30 and 50, with a minimum of five symptomatic uterine fibroids with a maximum diameter of 6 cm for the largest myoma, all intramural or subserous types, and uterine sizes smaller than 24 weeks of pregnancy. We excluded women with a history of prior surgeries, hypertension, heart or lung illness, bleeding disorders, anemia (hemoglobin (Hb) < 10 g %), chronic endocrine or metabolic diseases such as diabetes, obesity (body mass index > 30 kg/m^2^), or instances requiring intraoperative conversion of myomectomy to hysterectomy.

RETRACTED

### Sample size calculation

The sample size was adjusted by confidence interval = 95%, margin of error = 5%, and study's power = 80%. Therefore, the minimum sample size for each group was 60.

### Treatment protocol

We examined all eligible patients, took full clinical history, and ordered investigations like complete blood count and ultrasound. Then, the baseline data were collected including age, body mass index, baseline HB and HCT, previous cesarean section (CS), parity, and indications for CS. Patients were separated into three simultaneous groups using simple randomization produced by a computer program. Their assignments were made using sealed opaque envelops.

All patients underwent the operation by whether the Pfannenstiel or midline vertical incisions. During myomectomy, the patients received whether an injection of 30 IU of oxytocin in 500 ml of normal saline administrated during myomectomy with two ampules of distilled water which had the same color and shape of Ethamsylate and tranexamic acid before skin incision IV (group 1); received injections of 1 g of TA, 250 mg of Ethamsylate, and 110 ml of normal saline IV with an ampule of distilled water infused in 500 ml normal saline which had the same shape and color of oxytocin during myomectomy; (group 2); or received an injection of 110 ml of normal saline IV just before surgical incision with two ampules of distilled water infused in 500 ml normal saline which had the same shape and color of oxytocin; (group 3). All patients, care givers and providers and outcome assessors were blinded.

### Outcomes

The primary outcome was the amount of intraoperative blood loss. The secondary outcomes included the HB, and hematocrit (HCT) values, the change in towels and suction bottle weights, the need for blood and iron transfusion, the duration of operation and hospital stay, the need for hysterectomy, and postoperative fever.

### Statistical analysis

We used SPSS version 25, IBM, USA to perform the analysis after the recording of data. We presented the qualitative variables by both number (n) and percentage (%) while the quantitative data were described by mean and standard deviation. The statistical test of one-way ANOVA was applied to evaluate quantitative outcomes while the chi-squared test was used for the qualitative outcomes. The results were considered significant when *P* values < 0.05.

RETRACTED

## Results

### Baseline and general characteristics

Our multi-center randomized clinical trial represents a sample of 180 female patients. They were randomly allocated to three equal groups (60 patients in each group). The first was given oxytocin 30 IU during myomectomy, the second was given TA 1 g and ethamsylate 250 mg once before the skin incision, and the third was given normal saline 110 ml before the skin incision, (Fig. 1). There was a significant difference between groups regarding their age (*P* = 0.036). However, there were non-significant differences between groups regarding body mass index, parity, doing a previous cs, and their indications for CS. Nearly half of the patients had never undergone a CS previously (47.2%). Moreover, the most typical causes for being indicated CS were having a previous CS (8.9%), elderly primigravida (7.8%), and obstructed labor (6.7%). However, the minor causes were failed labor process (1.7%), rupture of membrane (1.1%), and having a uterine fibroid (1.1%), (Table 1).

**Fig. 1:** CONSORT 2010 flow diagram

**Table 1:** Baseline characteristics

	**Oxytocin**	**Tranexamic acid and ethamsylate**	**Saline**	***P* value**	
**Age (year)**	31.08 (4.22)	31.33 (3.82)	29.52 (4.37)	0.036	
**BMI [(kg/(m)**^**2**^**]**	26.87 (6.2)	27.18 (5.88)	27.17 (5.83)	0.984	
**Preoperative HB (g %)**	10.8 (0.77)	10.81 (0.83)	10.9 (0.84)	0.760	
**Preoperative HCT (%)**	32.38 (2.32)	32.41 (2.51)	32.79 (2.58)	0.604	
**Preoperative towel’s weight (mg)**	150	150	150	–	
**Preoperative suction bottle’s weight (mg)**	250	250	250	–	
**Previous CS**	Yes: 6 (10%) No: 54 (90%)	Yes: 3 (5%) No: 31 (51.6%) Missing: 26	NR	0.581	
**Parity**					
PG	15 (25%)	16 (26.7%)	20 (33.3%)	0.993	
P1	9 (15%)	9 (15%)	9 (15%)		
P2	15 (25%)	16 (26.7%)	11 (18.3%)		
P3	14 (23.3%)	13 (21.7%)	14 (23.3%)		
P4	2 (3.3%)	1 (1.7%)	1 (1.7%)		
P5	5 (8.3%)	5 (8.3%)	5 (8.3%)		
**Indication for CS**				Total	*P* value
Previous C.S	8 (13.3%)	4 (6.7%)	4 (6.7%)	16 (8.9%)	1
Elderly PG	5 (8.3%)	5 (8.3%)	4 (6.7%)	14 (7.8%)	
Obstructed labour	4 (6.7%)	4 (6.7%)	4 (6.7%)	12 (6.7%)	
CPD	4 (6.7%)	3 (5%)	4 (6.7%)	11 (6.1%)	
Occipitoposterior position	2 (3.3%)	4 (6.7%)	4 (6.7%)	10 (5.6%)	
Uterine rupture	2 (3.3%)	4 (6.7%)	3 (5%)	9 (5%)	
Breech	3 (5%)	3 (5%)	2 (3.3%)	8 (4.4%)	
DM	2 (3.3%)	2 (3.3%)	4 (6.7%)	8 (4.4%)	
Birth defects	2 (3.3%)	1 (1.7%)	4 (6.7%)	7 (3.9%)	
Precious baby	2 (3.3%)	4 (6.7%)	1 (1.7%)	7 (3.9%)	
1ry infertility	2 (3.3%)	2 (3.3%)	2 (3.3%)	6 (3.3%)	
Deflexed head	2 (3.3%)	2 (3.3%)	2 (3.3%)	6 (3.3%)	
Gestational diabetes	2 (3.3%)	2 (3.3%)	2 (3.3%)	6 (3.3%)	
Preeclampsia	2 (3.3%)	2 (3.3%)	2 (3.3%)	6 (3.3%)	
Triplet pregnancy	1 (1.7%)	2 (3.3%)	3 (5%)	6 (3.3%)	
Prolonged labour	1 (1.7%)	2 (3.3%)	2 (3.3%)	5 (2.8%)	
APH	1 (1.7%)	2 (3.3%)	1 (1.7%)	4 (2.2%)	
Cord around neck	1 (1.7%)	1 (1.7%)	2 (3.3%)	4 (2.2%)	
Cord prolapse	2 (3.3%)	1 (1.7%)	1 (1.7%)	4 (2.2)	
Fetal distress	2 (3.3%)	1 (1.7%)	1 (1.7%)	4 (2.2%)	
Footling presentation	2 (3.3%)	1 (1.7%)	1 (1.7%)	4 (2.2%)	
Large sized baby	1 (1.7%)	2 (3.3%)	1 (1.7%)	4 (2.2%)	
Placenta Previa	2 (3.3%)	1 (1.7%)	1 (1.7%)	4 (2.2%)	
Polyhydraminos	1 (1.7%)	2 (3.3%)	1 (1.7%)	4 (2.2%)	
Twins	1 (1.7%)	2 (3.3%)	1 (1.7%)	4 (2.2%)	
Failed Labor Progress	1 (1.7%)	1 (1.7%)	1 (1.7%)	3 (1.7%)	
ROM	1 (1.7%)	0	1 (1.7%)	2 (1.1%)	
Uterine Fibroid	1 (1.7%)	0	1 (1.7%)	2 (1.1%)	

Represents the baseline and general characteristics of the sample population, continuous values are presented as mean (SD), while dichotomous values are presented as number (percentage)

*BMI* Basal Metabolic Index, *HB* Hemoglobin, *HCT* Hematocrit, *CS* Cesarean Section, *PG* Primigravida, *CPD* Cephalopelvic disorder, *DM*; Diabetes Mellitus, *APH* Antepartum haemorrhage, *ROM* Rupture of membrane, and *NR* Not reported

Before the operation, we measured HB and HCV values for each patient, and they showed non-significant differences between groups as well (*P* = 0.760 and *P* = 0.604 for HB and HCT, respectively). Also, the preoperative towels' weights were 150 mg, and the preoperative suction bottle weight was 250 mg, (Table 1).

RETRACTED

### Primary outcome

#### Blood loss

There was a non-significant difference between groups regarding blood loss, with a mean of 666.25 ± 183.03 for oxytocin, 630.72 ± 145.83 for tranexamic acid and ethamsylate and 646.67 ± 168.92 for saline (*P* = 0.506), (Table 2).

**Table 2:** Primary and secondary outcomes

		**Oxytocin**	**Tranexamic acid and ethamsylate**	**Saline**	***P* value**
**Blood loss (ml)**	Mean (SD)	666.25 (183.03)	630.72 (145.83)	646.67 (168.92)	0.506
**Postoperative HB (g%)**	Mean (SD)	8.92 (1.25)	9.12 (1.23)	9.07 (1.33)	0.670
**Postoperative HCT (%)**	Mean (SD)	26.5 (4.81)	26.88 (3.92)	26.45 (4.53)	0.828
**Postoperative towels' weights (mg)**	Mean (SD)	509.25 (112.2)	496.87 (102.57)	505.72 (108.84)	0.811
**Postoperative suction bottle weight (mg)**	Mean (SD)	557 (83.39)	533.85 (77.49)	540.95 (84.02)	0.286
**Operative time (minutes)**	Mean (SD)	65.67 (19.95)	63.08 (18.39)	64.92 (20.51)	0.760
**Postoperative Hospital stay (days)**	Mean (SD)	2.3 (2.17)	2.33 (2.15)	2.27 (2.18)	0.986
**Postoperative wound infection**	Yes	12 (20%)	12 (20%)	12 (20%)	1
**Postoperative fever**	Yes	12 (20%)	14 (23.3%)	10 (16.7%)	0.659
**Need to hysterectomy**	Yes	0	0	0	–
**Intra or Postoperative blood transfusion**	Yes	13 (21.7%)	9 (15%)	12 (20%)	0.624
**Postoperative parenteral iron transfusion**	Yes	12 (20%)	13 (21.7%)	11 (18.3%)	0.901

Represents outcomes values among groups, continuous values are presented as mean (SD), while dichotomous values are presented as number (percentage)

*HB* Hemoglobin, and *HCT* Hematocrit

RETRACTED

### Secondary outcomes

#### HB and HCT values

After applying a paired t-test, each drug showed a significant decrease in HB and HCT levels compared to the baseline (*P* < 0.001). However, when using way ANOVA test comparing the postoperative and change values, all study drugs showed non-significant differences. For HB values, the differences were for postoperative and change values were non-significant (*P* = 0.670 and *P* = 0.677, respectively). Also, for HCT values, the differences for postoperative and changed values were non-significant (*P* = 0.828 and *P* = 0.554, respectively), (Tables 2, 3, 4).

**Table 3:** Mean differences for different secondary outcomes compared to the baseline

		**Oxytocin**	**Tranexamic acid and ethamsylate**	**Saline**
**HB (g%)**	Preoperative	10.8 (0.77)	10.81 (0.83)	10.9 (0.84)
	Postoperative	8.92 (1.25)	9.12 (1.23)	9.07 (1.33)
	Change	-1.88 (1.2)	-1.69 (1.1)	-1.83 (1.25)
	*P* value, 95% CI	*P* < 0.001	*P* < 0.001	*P* < 0.001
		95%CI (-2.19, -1.56)	95%CI (-1.97, -1.41)	95%CI (-2.15, -1.5)
**HCT (%)**	Preoperative	32.38 (2.31)	32.41 (2.51)	32.79 (2.58)
	Postoperative	26.5 (4.18)	26.88 (3.92)	26.45 (4.53)
	Change	-5.88 (4.05)	-5.53 (3.84)	-6.34 (4.38)
	*P* value, 95% CI	*P* < 0.001	*P* < 0.001	*P* < 0.001
		95%CI (-6.93, -4.83)	95%CI (-6.52, -4.54)	95%CI (-7.47, -5.21)
**Towels’ weight (mg)**	Preoperative	150	150	150
	Postoperative	509.25 (112.2)	496.87 (102.57)	505.72 (108.84)
	Change	359.25 (112.2)	346.86 (102.57)	355.72 (108.84)
	*P* value, 95% CI	*P* < 0.001	*P* < 0.001	*P* < 0.001
		95%CI (330.26, 388.24)	95%CI (320.37, 373.36)	95%CI (327.6, 383.83)
**Suction bottle weight (mg)**	Preoperative	250	250	250
	Postoperative	557 (83.89)	533.85 (77.49)	540.95 (84.02)
	Change	307 (83.89)	283.85 (77.49)	290.95 (84.02)
	*P* value, 95% CI	*P* < 0.001	*P* < 0.001	*P* < 0.001
		95%CI (285.33, 328.67)	95%CI (263.83, 303.87)	95%CI (269.25, 312.65)

Represents the mean difference of each drug value compared to the baseline value, continuous values are presented as mean (SD)

*HB* Hemoglobin, *HCT* Hematocrit, and *CI* Confidence Interval

**Table 4:** Change values of different outcomes

	**Oxytocin**	**Tranexamic acid and ethamsylate**	**Saline**	***P* value**
**HB change (g%)**	-1.88 (1.2)	-1.69 (1.1)	-1.83 (1.25)	0.677
**HCT change (%)**	-5.88 (4.05)	-5.53 (3.84)	-6.34 (4.38)	0.554
**Towels' weights (mg)**	359.25 (112.2)	346.87 (102.57)	355.72 (108.84)	0.811
**Suction bottle weight (mg)**	307 (83.89)	283.85 (77.49)	290.95 (84.02)	0.286

Represents the difference between the change values of different outcomes among groups, continuous values are presented as mean (SD)

*HB* Hemoglobin, and *HCT* Hematocrit

RETRACTED

#### Towels and suction bottle weight

After applying a paired t-test, each drug showed a significant increase in towels' weights and suction bottle weight compared to the baseline (*P* < 0.001). However, when applying one-way ANOVA comparing the postoperative and the change values, all study groups showed non-significant differences. The differences between towels' weight values were *P* = 0.811 for both postoperative and change values. Also, for suction bottle weight, the differences were *P* = 0.286 for both postoperative and change values, (Tables 2, 3, 4).

#### Other secondary outcomes

Applying the ANOVA test, all study outcomes showed non-significant differences between all groups including operative time (*P* = 0.760), hospital stay (*P* = 0.986), postoperative wound infection (*P* = 1), postoperative fever (*P* = 0.659), intra/postoperative blood transfusion (*P* = 0.624), and postoperative parenteral iron transfusion (*P* = 0.901). On the other hand, none of the patients from all groups needed a hysterectomy.

## Discussion

This RCT indicated that oxytocin and TA with ethamsylate had no significant value in lowering intraoperative blood loss compared with the placebo for abdominal myomectomy. Also, the changes in both HB and HCT values showed no significant differences between the three groups. Non-significant trends were observed for a reduction in operation time, intra/postoperative blood transfusion, hospital stay, postoperative fever, and wound infection.

Our results contrasted with a prior RCT conducted on the Egyptian population. They found that women assigned to get TA and ethamsylate instead of oxytocin experienced substantially less intraoperative blood loss during myomectomy [13]. However, the sample size in their RCT was small, as it was equal to half the sample size in our study.

Furthermore, two recent systematic reviews and meta-analyses found that prophylactic TA was associated with considerable decreases in total, intra, and postoperative blood loss compared to the placebo for women undergoing myomectomy [14]. According to dysfunctional uterine bleeding, the combination of TA and ethamsylate influenced the bleeding control. However, TA was better than ethamsylate for decreased blood loss and enhanced quality of life [15]. Additionally, TA and ethamsylate could considerably reduce blood loss during and following a cesarean section [16]. A similar finding was observed regarding oxytocin, as it was revealed that preventive oxytocin administration dramatically lowered intraoperative blood loss during abdominal myomectomy [10].

RETRACTED

Concerning HB and HCT levels, our study was in line with two previous analyses that showed that in comparison to the control group, preventive TA and oxytocin were linked to a considerable reduction in postoperative HB and HCT [8].

Despite that, a preventative TA was associated with a considerably shorter hospital stay following myomectomy in a prior study; there was no evident difference in the operating time and blood transfusion rate between the intervention and placebo, which is consistent with our findings [8].

All the perioperative therapies discussed above have self-limited adverse effects regarding safety outcomes. Although these events are discovered to be extremely low. TA is generally safe; however, intravenous TA is believed to raise the risk of thromboembolic and cardiovascular morbidities [17]. Also, uterotonic drugs such as oxytocin may cause hypertension, nausea, vomiting, and abdominal discomfort [18]. However, the participants in our study who received TA, ethamsylate, or oxytocin experienced no significant side effects.

Compared to GnRH analogs, the most common approach for lowering myomectomy bleeding, TA and ethamsylate, are less expensive [19]. Also, compared to vasopressin, TA and ethamsylate are safer and less costly. Some adverse effects have been associated with intraoperative vasopressin, including mistaken intravascular infiltration, hemorrhage at the puncture site, and brief elevation in blood pressure during injection [20].

### Limitations

The main limitation of this RCT is the scant number of published RCTs in this field. The amount of evidence that is now available on this topic is still insufficient to draw solid conclusions about the efficacy of the discussed therapies. Future research should compare prophylactic oxytocin against TA with ethamyslate among myomectomy patients pre- and post-operatively in additional multicenter, large-sized, and well-controlled RCTs.

## Conclusion

This RCT indicated that oxytocin and TA with ethamsylate had no significant value in lowering intraoperative blood loss compared with the placebo for abdominal myomectomy which opens a new question about the role of the use of the hemostatic drug during myomectomy especially in centers with limited resources and had higher rates. Additional studies are still required to verify our findings and examine the influence of myomectomy type and fibroid features on the amount of blood lost during myomectomy.

RETRACTED

## Data Availability

The datasets used and/or analyzed during the current study are not publicly available due to the confidentiality of participants' data and the difficulty of organizing the raw data to be suitable for publication; however, they are available from the corresponding author on reasonable request.
